RETRACTED

# UAV Communication Network Modeling and Energy Consumption Optimization Based on Routing Algorithm

**DOI:** 10.1155/2022/4782850

**Published:** 2022-06-28

**Authors:** Ran Zhuo, Shiqian Song, Yejun Xu

**Affiliations:** ^1^Fundamental Experimental Teaching Department, Nanjing University of Aeronautics and Astronautics, Nanjing, 211100 Jiangsu, China; ^2^Yangzhou Marine Electronic Instruments Institute, Yangzhou, 225101 Jiangsu, China

## Abstract

Topological information is provided, and research on the design of routing protocols for UAV self-assembling networks is conducted, in order to enable fleet communication transfer between UAVs and UAVs and enhance their communication transmission rate in the self-assembling network. A new routing protocol is proposed through greedy forwarding and peripheral forwarding of UAV self-assembling network communication data, UAV self-assembling network planarization processing, dynamic adjustment of routing mode based on topological information, and routing protocol decision content generation. The proposed network is described using stochastic geometry theory, with the UAV and building locations modeled as two independently distributed Poisson point processes and the building shape modeled as a rectangular body with height obeying the Rayleigh distribution. An estimated equation for typical user coverage is produced using this model. The simulation results show that the approximate expression matches with the simulation results with reduced computational complexity, which verifies the validity of the approximate analysis. By comparing it with the clustering-based routing protocol, it is concluded that the new routing protocol conditions for UAV self-assembly network can realize the communication transmission between UAVs and drones and further promote their communication transmission rate.

## 1. Introduction

The existing unmanned aerial vehicle (UAV) autonomous network is generated on the basis of Ad network, which can realize the centerless and self-organized communication transmission method without relying on ground communication equipment in practical applications. However, this network structure has no central node in the process of communication transmission, so each communication node is able to join and leave the network freely, which makes the communication capability of the UAV itself reduce and has the problem of drastic changes in network topology. Both for the security of communication data information and for the operation of the UAV itself, there is a certain negative impact. Therefore, to address this problem, this paper carries out research on the design of UAV self-assembling network routing protocols based on the introduction of topology information technology [1–3].

RETRACTED

Based on the topological information of UAV self-assembling network routing protocol design, UAV self-assembling network communication data greedy forwarding, and peripheral forwarding according to the communication transmission between UAV and UAV swarm, the communication data forwarding mode should be designed according to the actual situation, combined with the spatial characteristics of UAV in the process of operation; two forwarding modes are designed from two aspects, namely, greedy forwarding and peripheral forwarding [4–6]. The first one is greedy forwarding: in the UAV self-organizing network structure, the neighboring transmission node with the smallest spatial linear distance between the local neighbor table and the transmission target node is selected from the transmission node as the next data delivery node, and the node is also taken as the core node in the routing protocol. The overall flow diagram of greedy forwarding is shown in Figure 1.

Combined with the content shown in Figure 1, *X* is taken as the data packet that needs to be transmitted for communication, the dashed circle in Figure 1 indicates the communication coverage of UAV A, and the solid arc indicates the arc with a point *D* of the communication coverage of another UAV *B* as the center of the circle and the line segment *d* (*D*, *Y*) as the diameter [7]. When packet *X* receives the data that needs to be transmitted, then the lowest distance can be selected by means of a straight-line distance calculation between *Y* and *D*, and the node corresponding to the shortest distance can be used as the next greedy forwarding node. Combined with the forwarding process discussed above, the delivery of packets is completed. In practical applications, greedy forwarding only needs to obtain the spatial geographic information of neighboring UAVs to achieve the selection of communication transmission paths. The second type is peripheral forwarding: this forwarding method is applicable to the forwarding needs that are smaller than the straight-line distance between each node in the above greedy forwarding, so it can be regarded as a way of in-place forwarding. When the distance of communication data transmission is insufficient, the packets will encounter routing hole problem during transmission and thus cannot be carried out according to the above greedy forwarding method [8–10]. A right-hand rule for perimeter forwarding is established to prevent routing holes when UAVs are sent in a self-organizing network, and a sequence of traversal operations is completed in a clockwise direction, forming a polygon region in the process. In the process of transmission, the source node gives a decision based on the routing information in the neighbor table and completes the next communication packet forwarding. When the next node receives the packet, the above operation is repeated to find the best next transmission node and so on until the packet is transmitted to the UAV destination node to realize the forwarding of UAV packets in the self-organizing network [10].

RETRACTED

UAV self-organizing network is one of the typical applications of mobile self-organizing network in UAV field. With the characteristics of self-organization, mobility, topological dynamics, and high destructive resistance, UAV self-organizing network has a wide range of applications in both military and civilian fields, such as geological survey, rescue and disaster relief, regional reconnaissance, and unmanned cluster cooperative operations. The topology of UAV self-organizing networks is mainly divided into flat network structure and hierarchical network structure, and the hierarchical network structure is more suitable for UAV self-organizing networks of medium scale and above. In the hierarchical network structure, the network nodes are divided into several clusters, and each cluster has a cluster head node and several cluster member nodes, where the cluster head node is responsible for managing the other nodes in the cluster and communicating with the cluster head nodes of other clusters, and when the cluster member nodes need to communicate with other nodes, they first send messages to their cluster heads, and then, the cluster heads forward the messages to the destination nodes. Because of the open wireless communication environment and the flexible and changeable collaboration mode, the UAV self-assembled network is vulnerable to internal and external attacks in the process of constructing topology and establishing routes. In the process of network topology construction, the main security threats faced by UAV self-assembled networks include tampering attacks and impersonation attacks. If the integrity of topology construction messages is compromised, it will lead to wrong data being used for network topology construction, forming an invalid or inefficient topology structure [11–13]. The existing work on security protection of UAV self-assembling network mainly focuses on identity legitimacy verification, message confidentiality protection, message integrity protection, malicious node detection, and other areas when messages are transmitted between nodes after the network topology is established and lacks message security protection mechanisms for the process of network topology establishment, and the existing few security protection schemes for topology messages are applicable to the UAV self-assembling network with flat network structure and cannot be directly applied to the hierarchical network. The few existing security protection schemes for topology messages are all applicable to the UAV self-assembled network of flat network structure and cannot be directly applied to hierarchical network structure.

RETRACTED

This paper is organized such that Section 2 defines some related work.  Section 3 proposes the main methods of the study.  Section 3 also explains the methods of the proposed work.  Section 3.5 defines the experiment and analysis of the proposed work. Finally, the paper ends with a conclusion in Section 4.

## 2. Related Work

In this section, we define the UAV communication network modeling and UAV communication routing.

### 2.1. UAV Communication Network Modeling

The rise of diversified application services is accompanied by the proliferation of end-users, and the massive number of connections and differentiated network demands places greater demands on wireless communication network systems. With the advantages of high mobility, easy deployment, and low cost [14, 15], UAV-based network communication solutions have emerged and gradually attracted the attention of researchers, and more and more research has been conducted. Although UAV-based communication makes up for the shortcomings of current wireless network systems and can provide flexible, reliable, and on-demand communication network services for end devices, the energy consumption and endurance problems of UAVs and the differentiated ground service requirements make it possible to improve transmission efficiency, access efficiency, and computational efficiency from three aspects: UAV network location deployment, network connection establishment, and network service provision. The research on UAV-based energy-efficient communication strategies has become a major hot area of current research. This section first summarizes the existing research on UAV-based communication to improve transmission efficiency and achieve energy-efficient network dynamic location deployment; then, it introduces the existing research on how to improve access efficiency and achieve energy-efficient access of ground devices for the scenario of massive ground devices accessing the network. Finally, it focuses on data computation offloading services for the provision of UAV-based communication network services. A synopsis of existing research on how to ensure computational efficiency and implement energy-efficient computational offloading using UAVs is presented. We examine the inadequacies of existing solutions and conduct out follow-up work to address the existing issues [16, 17].

RETRACTED

After completing the deployment of UAV-based energy-efficient optimization, how to establish the network connection between ground terminal devices and UAV-based communication platform becomes the next issue to be considered, especially for the mass-connected IoT terminal devices, which are often in remote areas and have extremely high requirements for energy consumption, However, because of the disparity between the large number of ground terminal users and limited wireless network access resources, as well as UAV range time, reducing access network congestion and overload, improving access resource utilization and terminal device access success rate, increasing access efficiency, and realizing energy-efficient network connection establishment based on UAVs are a critical problem that requires immediate attention. It has attracted a lot of discussion and attention in academia and industry. According to the difference in the location of the triggering network connection establishment service, the research of energy-efficient network connection establishment can be divided into push-type and pull-up-type energy-efficient network connection establishment schemes to alleviate access congestion and improve access efficiency at the same time.

After completing the deployment of UAV-based energy-efficient optimization, the next issue to consider is how to establish network connections between ground terminal devices and UAV-based communication platforms. This is especially important for mass-connected IoT terminal devices, which are often in remote areas and have extremely high energy consumption requirements, so UAVs' flexible mobility makes them an important means of assisting in IoT network access. A crucial means of increasing capacity [18, 19]. However, the contradiction between the huge number of ground terminal users and limited wireless network access resources and UAV range time makes how to reduce access network congestion and overload, improve access resource utilization and terminal device access success rate, increase access efficiency, and realize energy-efficient network connection establishment based on UAVs an important problem that needs to be solved urgently and has attracted much discussion and attention in academia and industry. It has attracted a lot of discussion and attention in academia and industry. According to the difference in the location of the triggering network connection establishment service, the research of energy-efficient network connection establishment can be divided into push-type and pull-up-type energy-efficient network connection establishment schemes to alleviate access congestion and improve access efficiency at the same time. The UAV communication schematic is shown in Figure 2.

RETRACTED

### 2.2. UAV Communication Routing

With the increasingly widespread application of UAV self-assembly networks, domestic and foreign scholars have proposed a large number of UAV self-assembly network routing protocols; however, there is less research on the security protection mechanism of routing protocols, and if the integrity of information in the routing establishment process cannot be guaranteed, malicious information may be used to establish the network topology and routing path process, which leads to unstable network topology, inefficient routing, and other problems This can have a significant negative impact on network performance [20].

The routing protocols of UAV self-assembled networks can be split into two categories based on network topology: nonhierarchical routing protocols and hierarchical routing protocols. Among them, the nonhierarchical routing protocols are applicable to the planar network structure, in which all nodes in the network have equal status and have the function of forwarding and routing, and the existing classical protocols include on-demand distance vector routing, optimal link state routing protocol, dynamic source routing protocol, geolocation routing protocol GPSR, and secure routing algorithm of aerial self-assembling network based on geolocation integrated selection of the next hop. However, in complex mission scenarios, with the increase of the number of UAV nodes in UAV self-assembling networks, hierarchical routing protocols have become a hot spot for research in order to balance the UAV node load and improve the stability of the network. The existing classical hierarchical routing protocols mainly include lowest ID clustering algorithm with the unique identifier ID number of network nodes as a factor and mobility prediction-based clustering algorithm that considers node movement factors. Weight-based clustering algorithm uses node energy, node degree, distance between nodes, and node movement speed as measurement criterion for nodes to run for cluster head. The reliability-based clustering algorithm divides the clustered network with node energy, link retention rate, node degree, and communication volume as factors and adjusts the weight of each factor in the clustering process with the objectives of enhancing topology stability, saving energy, and improving service quality, respectively, to achieve network topology stability, reducing energy consumption or improving network service quality to the maximum extent. In the above hierarchical routing protocols, the formation of routes is built on the basis of building a hierarchical topology of the network, i.e., completing the clustering of network nodes [18].

RETRACTED

In UAV self-assembled network routing security protection mechanism, attackers may launch a sequence of malicious actions to disrupt the routing system by eavesdropping on the control information at the network layer, making UAV networks communicating through wireless media more vulnerable to attacks than cable networks. Exposed to the vulnerable wireless environment, the network information security transmission of wireless self-assembled networks must satisfy both the security of data communication and the security of routing protocols. Currently, several schemes have been proposed to protect the routing protocols of UAV self-assembled networks. Manel proposes security enhancement methods for AODV protocols to protect the security of route discovery phase information and routing error information. We found that there is less research on the security protection mechanism for hierarchical routing protocols, and there is an urgent need to design an efficient and lightweight security protection mechanism for hierarchical routing protocols to ensure the integrity of the topology construction information transmitted between nodes during the construction of the network topology and to avoid the formation of inefficient or invalid topologies due to malicious attacks or failures that cause erroneous information to be used in the topology construction process and have negative impact on the upper layer services. In terms of data integrity protection, blockchain is increasingly being utilized to preserve the integrity of information due to its traceability and tamper-evident qualities, in addition to the use of hash functions and digital signature technology. In response to the current problem of the lack of security protection mechanism of the hierarchical UAV self-organizing network routing protocol, this paper proposes a security protection scheme for routing messages in the hierarchical routing protocol of the UAV self-organizing network. The scheme can guarantee the integrity of the interaction messages between nodes in the topology establishment process of the hierarchical network structured UAV self-organized network. In the scheme, blockchain technology is used to store static topology messages and verify and ensure their integrity, while reducing the resource overhead of the proposed scheme.

## 3. Methods

In the method section, we discuss the model structure, antenna model, channel model, and channel model in detail.

### 3.1. Model Structure

A UAV wireless communication network in the 3D environment of a building is selected as the research object, and its system framework is shown in Figure 3. Firstly, consider buildings in cities, which are generally assumed to be rectangular in shape; their horizontal dimensions, heights, and orientations are random and mutually independent; and the central points constitute a uniform Poisson point process in the 2D plane with intensity *λB*.Assume that the distribution of the length*L*and width*W*of each building obeys specific probability density functions*f*_*L*_(*y*)and*f*_*W*_(*y*)with expectations which are*𝔼*[*L*]and*𝔼*[*W*]. The orientation angle of the building is denoted by *φ*, which is uniformly distributed on (0, 2*π*]. The height *h*_B_ of the building obeys the Rayleigh distribution, and its probability density function is

(1) $$\begin{array}{c} f_{H_{\text{B}}}\left(h_{\text{B}}\right)=\frac{h_{\text{B}}}{\sigma^{2}}e^{-\left(h_{\text{B}}^{2}/2\sigma^{2}\right)}. \end{array}$$

RETRACTED

### 3.2. Antenna Model

In order to compensate for the high road loss characteristics of millimeter wave, it is assumed that both UAV and user are assembled with uniform planar square array (UPA) to achieve directional beam assignment, and the antenna gain is a complex function defined by the antenna azimuth and elevation angles. Using beam alignment and tracking techniques, it is assumed that the antenna main flaps at the transmitter and receiver ends can be perfectly aligned to achieve the maximum power gain. In the azimuth plane, the half-power beamwidths of the UAV antenna and the user antenna can be denoted as *θ*^*a*^_A_ and *θ*^*a*^_U_, respectively, and the corresponding half-power beamwidths in the elevation plane are *θ*^*e*^_A_ and *θ*^*e*^_U_, respectively, and the main flap gains of the UAV and user antennas are *G*_A_ and *G*_U_, and the side flap gains are *G*_A_ and *G*_U_, respectively, and the probability distribution function of the total antenna gain *G* received at the receiving end is

(2) $$\begin{array}{c} G=\left\{\begin{array}{c} G_{\text{A}}G_{\text{U}},\zeta_{1}=p_{1}p_{2},\\ g_{\text{A}}G_{\text{U}},\zeta_{2}=\left(1-p_{1}\right)p_{2},\\ G_{\text{A}}g_{\text{U}},\zeta_{3}=p_{1}\left(1-p_{2}\right),\\ {\text{g}}_{\text{A}}g_{\text{U}},\zeta_{4}=\left(1-p_{1}\right)\left(1-p_{2}\right). \end{array}\right. \end{array}$$

*ζ*_*i*_ (*i* = 1, 2, 3, 4) is the distribution probability of *G*; *p*_1_ and *p*_2_ are the probabilities of antenna main flap alignment at the UAV side and the user side, respectively. The subscript *c* ∈ {*A*, *U*} is used to denote the UAV side and user side.

(3) $$\begin{array}{c} p_{1}\&=\frac{\theta_{\text{A}}^{a}}{2\pi }\frac{\theta_{\text{A}}^{e}}{\pi },\\ p_{2}\&=\frac{\theta_{\text{U}}^{a}}{2\pi }\frac{\theta_{\text{U}}^{e}}{\pi },\\ G_{c}\&=N_{c},\;c\in \left\{\text{A},\text{U}\right\},\\ g_{c}\&=\frac{\sqrt{N_{c}}-\left(\sqrt{3}/2\pi \right)N_{c}\sin\left(\sqrt{3}/2\sqrt{N_{c}}\right)}{\sqrt{N_{c}}-\left(\sqrt{3}/2\pi \right)\sin\left(\sqrt{3}/2\sqrt{N_{c}}\right)},\;c\in \left\{\text{A},\text{U}\right\}. \end{array}$$

RETRACTED

### 3.3. Channel Model

The large-scale fading term and the small-scale fading term of the millimeter-wave channel are considered comprehensively. The large-scale fading caused by path loss can be expressed as (*d*) = *d* − *α*, where *d* is the distance from the UAV to the user and *α* is the path loss index of the channel. Assumption 1 implies that the structures along the millimeter-wave communication link entirely block the millimeter-wave signal; i.e., the millimeter wave cannot pass through. For Assumption 2, the small-scale fading channel is a *Nakagami* channel, and the channel power gain is a gamma random variable *z* with probability density function

(4) $$\begin{array}{c} f_{Z}\left(z\right)=\frac{m^{m}z^{m-1}}{\Gamma \left(m\right)}\exp\left(-mz\right), \end{array}$$

where *m* is the shape factor of Nakagami channel and Γ(*m*) is the gamma function of *m*.

### 3.4. Performance Optimization

Since both the UAV and the user are equipped with directional antennas in the system, the ambient noise in the system is negligible compared to the power of the interference. Therefore, only the signal-to-interference ratio (SIR) received at the user side is considered as a parameter for performance evaluation. Under the 3D network model and the corresponding assumptions, the SIR received by a typical user in the downlink can be expressed as

(5) $$\begin{array}{c} \text{SIR}=\frac{G_{1}z_{0}{\left[{\left(h_{\text{A}}-h_{\text{U}}\right)}^{2}+R_{0}^{2}\right]}^{-\left(\alpha /2\right)}}{\sum_{i\in \psi \setminus 0}\;G_{i}z_{i}{\left[{\left(h_{\text{A}}-h_{\text{U}}\right)}^{2}+R_{i}^{2}\right]}^{-\left(\alpha /2\right)}S_{i}}, \end{array}$$

where *R*_0_ and *R*_*i*_ are the horizontal distances from the typical user to the serving drone and the interfering drone *i*, respectively; *S*_*i*_ is the total penetration power loss caused by the buildings on the *OX*_*i*_ link; and *z*_0_ and *z*_*i*_ are the small-scale fading terms of the serving link and the interfering link, respectively. Interference can be expressed as

(6) $$\begin{array}{c} I=\underset{i\in \psi \setminus }{\sum }\;G_{i}z_{i}{\left[{\left(h_{\text{A}}-h_{\text{U}}\right)}^{2}+R_{i}^{2}\right]}^{-\left(\alpha /2\right)}S_{i}. \end{array}$$

Then, the coverage can be further expressed as

(7) $$\begin{array}{c} {\mathbb{P}}_{\text{COV}}\left(T\right)=\&\mathbb{P}\left(\text{SIR}>T\right)=E_{x}\left[P\left(\text{SIR}>T\right)\right]=\int_{0}^{\infty }\mathbb{P}\left(\text{SIR}>T\left|R_{0}=x\right.\right)f_{R}\left(x\right)\text{d}x=\int_{0}^{\infty }\;\mathbb{P}\left\{z_{0}>TG_{1}^{-1}{\left[{\left(h_{\text{A}}-h_{\text{U}}\right)}^{2}+x^{2}\right]}^{a/2}I\right\}f_{R}\left(x\right)\text{d}x, \end{array}$$

where *f*_*R*_(*x*) is the probability density function of the distance from a typical user to the unobstructed and closest UAV and *T* is the signal-to-media ratio threshold at the receiver side that can correctly demodulate the signal. Since the small-scale fading channel from the UAV to the user is a *Nakagami* channel, i.e., the power gain *z*_0_ is a random variable obeying a gamma distribution.

RETRACTED

### 3.5. Air-to-Ground Channel Modeling

Figure 4 depicts the basic model of the UAV network. This UAV network consists of an observation UAV *A*, a relay UAV *R* based on the decode-and-forward collaboration approach, and a base station *B*. The UAV *A* flies over the observation area and collects observation information, and since the direct connection between UAV *A* and base station *B* is blocked by obstacles such as mountains or buildings, the collected information needs to be delivered to base station *B* through the relay UAV *R*. The UAVs are set to be configured with an unlimited size data buffer, and the data that UAV *A* or *R* cannot deliver to the target in time due to the channel capacity limitation that can be cached in the buffer. To facilitate the analysis, a 3D Cartesian coordinate system scenario is considered in this chapter. UAV *A* makes a circular motion of radius *r* over the observation area; it flies at a fixed altitude *H* and has a fixed velocity *V*. Therefore, the period of UAV *A* flying for one week can be derived.

(8) $$\begin{array}{c} T_{0}=\frac{2\pi r}{V_{0}}. \end{array}$$

Since the UAV often flies at high altitude, the flight height *H* of the UAV is much greater than the height of the base station *B*. Therefore, the height of the base station *B* can be ignored in the analysis. It can be obtained that the coordinates of *B* can be expressed as *O* (0, 0, 0), and the horizontal distance from base station *B* to the center of UAV *A*'s flight trajectory circle *O*′ is *D*. Therefore, the coordinates of the center of *A*'s flight trajectory circle can be expressed as *O*′ (*D*, 0, *H*). The relay UAV *R* is free to fly in the space between *A* and *B*, but the flight altitude of *R* is always kept the same as that of *A*, which is *H*. Meanwhile, the maximum flight speed of the UAV *R* is limited to dagger. The overall operation time of the relay UAV is assumed to be *T*, while the takeoff and landing phases of the UAV are not considered. Therefore, at time *t*, the time-varying coordinates of UAV *A* can be expressed as *X*_*A*_(*t*), *Y*_*A*_(*t*), *H*), while the time-varying coordinates of UAV*R*can be expressed as, where*t*takes values in the range [*O*, *T*]. To facilitate the calculation, the operation time *T* of the relay UAV is evenly divided into *N* equal parts, and each time slot can be denoted as *t*_0_ = *T*/*N*. When *N* is taken large enough, the positions of the UAV *A* and the relay *R* can be regarded as fixed in each time slot TO. Due to the good mobility of UAVs, the communication links of UAV networks can avoid obstacles in most cases, so it is assumed that the communication channels from *A* to *R* and *R* to *B* are mainly composed of line-of-sight channels. In addition, the Doppler effect is assumed to be perfectly compensated at both the receiving end *R* and *B* and does not need to be considered. The relay UAV *R* operates in full duplex mode and uses frequency division duplex technology, where the bandwidth of the transmit channel is equal to the bandwidth of the receive channel. In this chapter, it is assumed that the transmit power of all UAVs is certain, as

(9) $$\begin{array}{c} P_{A}=P_{R}=P_{0}, \end{array}$$

where *P*_*A*_ denotes the transmit power of the observation UAV *A*, *P*_*R*_ denotes the transmit power of the relay UAV *R*, and *P*_*O*_ denotes the fixed transmit power, which is a constant. In addition, the noise power is also assumed to be constant, as

(10) $$\begin{array}{c} P_{\text{N},A}=P_{\text{N},R}=P_{\text{N},B}=P_{\text{N}}, \end{array}$$

where *P*_N,*A*_ denotes the noise power at UAV *A*, *P*_N,*R*_ denotes the noise power at relay UAV *R*, *P*_N,*B*_ denotes the noise power at the base station, and *P*_N_ denotes the fixed noise power, which is a constant. Since the bandwidth of the communication channel is fixed in this UAV network, it is known that the performance of the communication link is related to the signal-to-noise ratio at the receiving end according to the Shannon formula, according to the free-space path loss model.

RETRACTED

The air-to-ground channel for UAV-based communication can be divided into two parts: LoS and non-line of sight. LoS communication is the wireless signal propagating in a straight line between the transmitter and the receiver with no obstacle occlusion *W*. NLoS communication is the wireless signal propagating between the transmitter and the receiving end which propagates with obstacle occlusion*W*. Take the Makoto city environment as an example, the air-to-ground channel of the UAV-based communication platform. Suppose the coordinates of a certain UAV are (*x*_*u*_, *y*_*u*_, *h*) and the coordinates where the user communicating with this UAV is located are (*x*_*g*_, *y*_*g*_, 0). When the wireless signal propagates in free space, the signal does not undergo the process of scattering, refraction, and diffraction, nor is it absorbed, and the path loss of the channel obeys the Gaussian distribution *N£*represents one of two channel types LoS and NLoS, i.e., ugly*E* ∈ {Los, NLoS}air-to-ground channel of a UAV-based communication platform. The path loss (in dB) in the LoS link and NLoS link cases is

(11) $$\begin{array}{c} L_{\text{LoS}}=L_{\text{FS}}+\eta_{\text{LoS}},\\ L_{\text{NLoS}}=L_{\text{FS}}+\eta_{\text{NLoS}}. \end{array}$$

The wireless signal propagation of the UAV-based communication platform in the urban environment is shown in Figure 5. The flight energy consumption of UAVs has a significant impact on the UAV endurance and greatly affects the efficiency of UAV-based communication. In simple terms, the flight energy consumption of UAV is related to its load as well as flight speed, and some related studies have modeled the energy consumption of UAVs simply as a model related to the mass and flight speed of UAVs [8-*u*]. Assume that the flight time of the UAV is *r* and the flight speed at moment *f* is *v*(*r*). The simple flight energy consumption model of the drone is

(12) $$\begin{array}{c} L_{\text{FS}}={\left(\frac{4\pi df}{c}\right)}^{2}, \end{array}$$

where *M* is the mass of the UAV. Although the simple energy consumption model is generally applied to the energy consumption model of UAVs, however, different types of UAVs are constructed differently and have different power systems, so the energy consumption models of different types of UAVs need to be considered. In this paper, the energy consumption models of fixed-wing UAVs and rotary-wing UAVs are introduced, respectively.

## 4. Experiments and Results

### 4.1. Experimental Setup

After completing the theoretical design of the topology-based routing protocol, the following comparison experiments are conducted to investigate the performance of the routing protocol in practical applications: the topology-based routing protocol and the cluster-based routing protocol proposed in this paper are introduced into two UAV devices of identical models and performance. In order to evaluate the performance of the two routing protocols in the UAV self-assembly network, an NS2 simulation device is installed in the Cygwin environment. The device is written in C++ using Otcl, and it is applied to the experimental environment of this paper to realize the simulation of UAV self-assembly network. The experimental environment built on the basis of this device contains a total of seven layers of network structure, whose corresponding TCP/IP relations are shown in Table 1. The hardware environment is shown in Table 2.

RETRACTED

According to the contents in Table 1, after clarifying the correspondence between the UAV self-assembled network structure and TCP/IP, the communication transmission rate of each hierarchical structure of the self-assembled network is calculated under the transmission conditions of the two routing protocols, and its calculation formula is as follows:

(13) $$\begin{array}{c} V=\frac{M\cdot \chi }{s}\log_{2}K. \end{array}$$

*V* denotes the communication transmission rate of each hierarchical structure of the UAV self-assembled network; *M* denotes the total amount of communication data generated in the communication process between UAVs; denotes the baud rate of data in the transmission process; *s* denotes the transmission time of data in each hierarchical structure; and *K* denotes the effective discrete value of communication data. The communication transmission rate of each level of the UAV self-assembly network under the two routing protocols is calculated.

### 4.2. Experimental Results and Analysis

To facilitate the comparison of the application performance of the two routing protocols, the calculated experimental results are recorded as shown in Table 3.*K* is denoted as the effective discrete value of the communication data. The communication transmission rate of the UAV self-assembled network at the starting level of the two routing protocols is calculated.

Therefore, the results obtained from the above experiments prove that the communication transmission rate of the seven levels of the UAV self-assembly network exceeds 12.00 Mbit/s under the conditions of the routing protocol in this paper; the highest communication transmission rate of the seven levels of the UAV self-assembly network is only 2.25 Mbit/s under the conditions of the routing protocol based on clustering. Therefore, the above experimental results prove that the routing protocol designed in this paper can achieve the communication transmission between UAVs and UAVs and achieve the application effect of efficient information transmission after the introduction of topology information technology.

Figure 6 shows the theoretical results and simulation results with good approximation. As the number of antenna array subunits equipped with UAV increases, the coverage of users corresponding to the same SIR threshold T also increases. This is due to the increase in the number of antenna arrays at the UAV end, which makes the antenna gain at the transmitting end larger, and the total gain of the useful signal received at the receiving end also increases, although the signal gain of the interfering UAV also increases, but because the main flap width of the directional antenna is narrow and randomly pointing, when the number of antenna arrays increases from 4 to 32, the probability of the main flap beam alignment between the transmitting end of the interfering UAV and the receiving end of the downlink user. Because the probability of the interference drone transmitter's primary flap beam alignment with the downlink user receiver drops from5.8 × 10^−3^to7.2 × 10^−4^, the impact of interference gain on user coverage performance is substantially smaller than that of usable signal gain. In addition, it can be seen from Figure 6 that when the threshold *T* of SIR is taken as 0 dB, the coverage rates at different numbers of antenna arrays are close to 1. This indicates that the number of antenna arrays of UAVs deployed in the area with lower quality of service requirements (i.e., lower SIR threshold) can be reduced, which can reduce the operator cost without affecting the system performance. And when the threshold of SIR is equal to 10 dB, the coverage rates corresponding to different antenna array numbers show significant differences, and the systems with antenna array numbers of 4 and 8 only correspond to coverage rates of 0.6 and 0.8. Therefore, in order to meet the areas with higher quality of service requirements, the number of antenna arrays of UAV-carrying antennas should be no less than 16.

RETRACTED

## 5. Conclusion

We conduct research on the design of their routing protocols in this paper, based on clarifying the operation mechanism of UAV self-assembling networks. We also incorporate topological information into the research process to achieve dynamic routing technique adjustment. When the routing protocol proposed in this paper is applied to the actual UAV self-assembling network, the routing mode can be dynamically adjusted based on the specific needs of communication transmission, allowing the routing mode to be dynamically adjusted to provide the required conditions for different transmissions and achieving an overall improvement in communication transmission rate. However, there are still many problems that need to be explored in the research process, such as the uncertainty of the motion law of the transmission nodes in the UAV self-assembling network; the transmission process should also be combined with a variety of motion models for improvement. As a result, in-depth research will be undertaken in the future to address the aforementioned issues, with the goal of boosting the routing protocol's perfection.

RETRACTED

## Figures and Tables

**Figure 1:** UAV self-organizing network communication data forwarding process diagram.

**Figure 2:** UAV communication schematic.

**Figure 3:** Model architecture.

**Figure 4:** The basic model of the UAV network.

**Figure 5:** UAV-based wireless signal propagation for communication platforms in urban environments.

**Figure 6:** Coverage with different numbers of antenna arrays.

**Table 1:** UAV self-assembling network structure and TCP/IP correspondence in the experimental environment.

Self-organizing network architecture	TCP architecture	IP architecture
Application layer	Application layer	Application layer
Representation layer	Application layer	Application layer
Session layer	Application layer	Application layer
Transport layer	Proxy layer	Transport layer
Network layer	Proxy layer	Network layer
Link layer	Nodes and connections	Physical layer
Physical layer	Nodes and connections	Physical layer

**Table 2:** Experimental hardware environment.

Operating system	Windows 10
CPU	Intel(R) Core(TM) i5-9400F CPU @ 2.90 GHz
Memory	8.00GB (RAM)

**Table 3:** Communication transmission rate of each hierarchy of UAV network.

Hierarchy	This article routing protocol V value	Cluster-based routing protocol
Application layer	12.26 Mbit/s	1.23 Mbit/s
Representation layer	15.26 Mbit/s	1.20 Mbit/s
Session layer	18.26 Mbit/s	1.02 Mbit/s
Transport layer	11.23 Mbit/s	1.23 Mbit/s
Network layer	15.26 Mbit/s	2.25 Mbit/s
Link layer	13.14 Mbit/s	1.85 Mbit/s
Physical layer	15.36 Mbit/s	1.67 Mbit/s

## Data Availability

The datasets used during the current study are available from the corresponding author on reasonable request.
